The article "Circulating FoxP3+ Regulatory T and Interleukin17-Producing Th17 Cells Actively Influence HBV Clearance in De Novo Hepatitis B Virus Infected Patients after Orthotopic Liver Transplantation" was retracted in 2019. Reasons: missing or withdrawn patient consent; ethical violations by an author; concerns about the data.

# Circulating FoxP3+ Regulatory T and Interleukin17-Producing Th17 Cells Actively Influence HBV Clearance in *De Novo* Hepatitis B Virus Infected Patients after Orthotopic Liver Transplantation

**DOI:** 10.1371/journal.pone.0137881

**Published:** 2015-09-14

**Authors:** Yinjie Gao, Min Zhang, Jin Li, Mei Yang, Yuan Liu, Xiaodong Guo, Hanwei Li, Zhenwen Liu, Jingmin Zhao

**Affiliations:** 1 Liver Transplantation and Research Center, 302 Military Hospital, Beijing, China; 2 Department of Infectious Diseases, Medical School of Chinese PLA, Beijing, China; 3 Department of Pathology and Hepatology, 302 Military Hospital, Beijing, China; 4 liver cirrhosis and Research Center, 302 Military Hospital, Beijing, China; CRCL-INSERM, FRANCE

## Abstract

**Objective:**

To longitudinally investigate the role of FoxP3+ Regulatory T cells (Treg) and interleukin17-producing T helper 17 cells (Th17) in De Novo Hepatitis B Virus infection after orthotopic Liver Transplantation (DNHB-OLT), and analyze the possible correlation between these cells and HBV clearance of the disease.

**Methods:**

We enrolled 12 control cases after orthotopic Liver Transplantation (OLT) and 24 patients, including 12 diagnosed with DNHB-OLT and 12 diagnosed with Acute Hepatitis B Virus infection (AHB), into the study from the liver transplantation and research center at Beijing 302 Hospital. Flow cytometry was used to detect the frequencies of Treg and Th17, and ELISA was applied to detect the concentration of IL6, IL22, TGF-β and IL2 in peripheral blood. We also measured the gene expression level by real time-quantitative PCR and protein expression using immunohistochemistry and western-blot. Furthermore, we divided DNHB-OLT patients into the clearance and non-clearance groups and examined longitudinally Th17, Treg cells at different times.

**Results:**

The percentage of Treg cells, expression of FoxP3 mRNA and related anti-inflammatory cytokines such as IL2 and TGF-β1 in the DNHB-OLT group were significantly higher than that in the AHB and OLT groups. The percentage of Th17 cells, expression of RORγt mRNA and related pro-inflammatory cytokines such as IL17 and IL22 in the DNHB-OLT group were significantly lower than that in the AHB group, but the levels of these cytokines are very similar to the OLT group. The ratios of Treg to Th17 in the DNHB-OLT group were significantly higher than that in the OLT and AHB groups. Treg frequencies significantly correlated with HBV DNA, whereas IL17 frequencies didn’t significantly correlate with ALT. In DNHB-OLT patients, the clearance group was accompanied by a rapid increase in the Th17 cells during the first 4^th^ week and afterwards continuously decrease to the control group, together with a continuously decrease in Treg cells from the onset time point, which lead to a significant reduction in the ratios of Treg to Th17. The non-clearance group was accompanied by an increase in the Treg cells during the first 4^th^ week and afterwards sharply decrease, together with a relatively stable and unchanged Th17 cells, which lead to a significant change in the ratios. In addition, compared to clearance group, the ratios of Treg to Th17 in non-clearance group were significantly higher at the onset point, 4^th^ and 12^th^ week, but no difference at 24^th^ week.

The article "Circulating FoxP3+ Regulatory T and Interleukin17-Producing Th17 Cells Actively Influence HBV Clearance in De Novo Hepatitis B Virus Infected Patients after Orthotopic Liver Transplantation" was retracted in 2019. Reasons: missing or withdrawn patient consent; ethical violations by an author; concerns about the data.

**Conclusion:**

DNHB-OLT patients possessed a favorable Treg differentiation environment, accompanied by a sustained higher preferentially Treg frequencies and up-regulation of related anti-inflammatory cytokines. The immune imbalance of the ratios between Treg and Th17 existed in DNHB-OLT patients. The changes of the ratios during the DNHB-OLT events were associated with HBV clearance, which suppressed immune inflammation reaction as well as inhibited ability of specific HBV clearance and led to immune escape and chronicity.

## Introduction

Liver obtained from hepatitis B surface antigen-negative (HBsAg-)/ hepatitis B core antibody-positive (HBcAb+) donors are increasingly used in many transplant centers because of the disparity between the liver allograft supply and the demand [1]. This practice varies with the regional incidence of hepatitis B virus (HBV), and such donors represent 3% to 6% of the donor pool in the United States, 8% to 15% of the donor pool in Europe, and 50% to 55% of the donor pool in Asia [2, 3]. However, the persistent of covalently closed circular DNA (cccDNA), which has been reported in HBsAg-/HBcAb+ donors, serves as original template for viral replication and plays an important role for virus reaction after transplant [4]. Using these donors, the rate of De Novo Hepatitis B Virus Infection after orthotopic Liver Transplantation (DNHB-OLT), which is defined as seroconversion from HBsAg- status to HBsAg+ status in recipients after organ transplantation, has reached up to 75% to 80% in HBsAg-/HBcAb- recipients and 5% to 10% in HBcAb+/hepatitis B surface antibody-positive (HBsAb+) without any prophylaxis [5]. Among HBV infection in adults, up to 90% of healthy population demonstrates self-limited infection, and most of them can be cleared by the host spontaneously and expresses itself as acute hepatitis B (AHB) infection [6]. However, 40% of DNHB-OLT appears chronicity [7, 8]. The outcomes after infection are significantly different between AHB and DNHB-OLT. HBV is not directly cytopathic and the hepatocellular injury caused by HBV infection is predominantly immune-mediated [9, 10]. HBV antigens induce cell-mediated immune responses, especially multispecific antiviral helper T cells (Th), and cytotoxic T lymphocytes (CTL) responses are essential for the clearance of viral infection from the liver [11]. Appropriate immune response can lead to viral clearance and recovery; whereas excess immune response can lead to liver failure and inadequate immune response will result in sustained HBV infection [12, 13].

The article "Circulating FoxP3+ Regulatory T and Interleukin17-Producing Th17 Cells Actively Influence HBV Clearance in De Novo Hepatitis B Virus Infected Patients after Orthotopic Liver Transplantation" was retracted in 2019. Reasons: missing or withdrawn patient consent; ethical violations by an author; concerns about the data.

CD4+CD25+Foxp3+ regulatory T cells (Treg), which comprise about 5–10% of the total CD4+ helper T cells, play an anti-inflammatory role mainly through contact dependent suppressing proliferation, cytokine production and cytotoxic activity of naïve and antigen-specific CD4+ and CD8+ effector T cells, and also are able to interfere with the activity of antigen-presenting cells as well as B cells [14]. Studies addressing the role of Treg in HBV infection mostly rely on correlation of Treg frequencies in peripheral blood of patients with different disease stages and have been somewhat contradictory [15, 16]. Thus we supposed Treg cells to be a ‘dual-edged’ sword during HBV infection for being detrimental to facilitate HBV escape and being protective to prevent immune-mediated liver injury.

Conversely, T helper 17 (Th17) cells, another newly identified subset of CD4+ cells with retinoid orphan nuclear receptor γt (RORγt) as the specific transcriptional factor, have also been involved in the pathogenesis of HBV infection [17, 18]. In contrast to Treg, Th17 cells induce strong inflammation response in autoimmune and infectious diseases through several key pro-inflammatory cytokines such as IL17, IL22, IL6, IL23, and tumor necrosis factor-a (TNF-a). Moreover, IL17 has been characterized as a major effector cytokine of Th17 and can recruit inflammatory cells into the liver and directly activate the hepatic natural immunity system to release cytokines that aggravate chronic inflammation and liver fibrosis [19]. Foxp3+Tregs and Th17 cells are closely associated with each other. Both of them require transforming growth factor (TGF-β) on development pathways [20] and accumulating data suggest the plasticity of Treg and Th17 cells under certain cytokine conditions. For example, Treg cells can be converted to IL17-expressing Th17 cells in response to IL6 and IL21, whereas Th17 cells can give a rise to Th1 or Th2 cells in the presence of IL12 or IL4, respectively [21].

Overall, Treg cells can suppress inflammation by secretion of immunosuppressive cytokines, whereas Th17 cells enhance inflammation of tissue through secretion of pro-inflammatory cytokines. The balance between Treg and Th17 cells might be crucial for immune homeostasis [22]. Recently, several research groups have demonstrated the imbalance of Treg/Th17 in HBV-associated patients including CHB [23], ACLF [24], and liver cirrhosis [25]. However, whether and how this imbalance influences the progression of AHB is still not clearly studied, especially without available information regarding the role of these two types of cells in DNHB-OLT. To address these issues, we designed this study to determine the frequencies and associated cytokines of Treg and Th17 cells in patients with DNHB-OLT, and to investigated the possible relationship of Treg/Th17 ratio with the disease progression and outcome in DNHB-OLT patients.

The article "Circulating FoxP3+ Regulatory T and Interleukin17-Producing Th17 Cells Actively Influence HBV Clearance in De Novo Hepatitis B Virus Infected Patients after Orthotopic Liver Transplantation" was retracted in 2019. Reasons: missing or withdrawn patient consent; ethical violations by an author; concerns about the data.

## Methods

### Patients

Twelve DNHB-OLT patients from June 2008 to June 2013 were enrolled into this study in the Department of Internal Transplantation of Beijing 302 Hospital. All the preoperative receptions were HBsAg-/HBcAb- and there were no HBV-related diseases and HCC. The liver donors were all HBsAg-/HBcAb+. No Hepatitis B immunoglobulin (HBIG) or nucleosides analog were applied for prevention during and after the transplantation. Most of the patients underwent induction with methylprednisolone, which was followed by tacrolimus and mycophenolate mofetil. DNHB-OLT was defined as the presence of one or more of the following parameters at any time after transplantation: HBsAg positivity, detectability of serum HBV DNA or hepatic covalently closed circular DNA [26]. The treatment of DNHB-OLT was initiated with Lamivudine (LAM) immediately and varied with the basis of HBV DNA loads, the availability of antiviral medications and renal function. The immunosuppression protocol was not modified because of the presence of de novo HBV. The disease control group with similar gender and age distribution to DNHB-OLT group was composed of 12 AHB patients, which was diagnosed with high serum titer of HBsAg and HBcAb of the immunoglobulin M (IgM) and acute onset elevation of serum ALT levels, excluding other origins of acute hepatitis, and with confirmed absence of HBsAg six months before admission (They all had negative results for serum HBsAg test). No patients received any antiviral or immunomodulatory therapy in the AHB group. In addition, the healthy control consisted of 12cases after orthotopic Liver Transplantation (OLT) with similar gender and age distribution to the two patients groups. There was no significant difference in the serum of the concentration of tacrolimus (FK506) and the time of follow up after liver transplantation between the DNHB-OLT group and OLT group. The clinical and pathological features in different groups were shown in Table 1. Venous blood samples were collected from the 24 patients when diagnosed (the onset point) and subsequently in DNHB-OLT groups on 4^th^, 12^th^, 24^th^ week (the end point) respectively. Liver biopsies were obtained from patients in AHB and DNHB-OLT groups for pathological evaluation once HBsAg positive was detected.

The article "Circulating FoxP3+ Regulatory T and Interleukin17-Producing Th17 Cells Actively Influence HBV Clearance in De Novo Hepatitis B Virus Infected Patients after Orthotopic Liver Transplantation" was retracted in 2019. Reasons: missing or withdrawn patient consent; ethical violations by an author; concerns about the data.

**Table 1:** Clinical characteristics in different groups. NA, not applicable; ALT, Alanine aminotransferase; Normal values: ALT, 0–40U/L; Acute Hepatitis B Virus (AHB), De Novo Hepatitis B Virus after Orthotopic Liver Transplantation (DNHB-OLT), Control cases after orthotopic liver transplantation (OLT)

	OLT	AHB	DNHB-OLT
Number (n)	12	12	12
Age (years)	42.3±9.2	38.4±13.2	41.8±10.3
Gender (male/female)	10/2	10/2	10/2
ALT (U/L)	27.3±14.2	433.2±57.1	186.9±43.8
HBV DNA (Log 10IU/mL)	NA	6.7±0.2	7.2±0.2
HBeAg (positive/negative)	NA	7/5	9/3
FK506 (ng/mL)	3.9±1.1	NA	4.1±0.7
Time after OLT (y)	31.7±5.3	NA	29.4±7.6

The written informed consents were obtained from all patients for liver biopsy and their clinical records to be used in this study, and their information was anonymized and de-identified prior to analysis. The study protocol was approved by the Medical Ethics Committee of the 302 Hospital, Beijing, China, and adhered to the Declaration of Helsinki. Organ donation was conducted legally, following local regulations. None of the transplant donors were from a vulnerable population or were subject to coercion.

### Flow cytometry to detect FoxP3+Treg and IL17-producing Th17 cells frequencies in peripheral blood

PerCP-conjugated Mouse anti-Human CD3 (Cat. #347344), FITC-conjugated Mouse anti-Human CD4 (Cat. #555346), APC-Cy7-conjugated Mouse Anti-Human CD25 (Cat. #557753), PE-conjugated Mouse anti-Human FoxP3 (Cat. #560046), PE-conjugated Mouse anti-Human IL17A (Cat. #560436) and Cytofix/Cytoperm Fixation/Permeabilization Solution Kit (Cat. #554714) were purchased from BD PharMingen (San Jose, CA, USA).

For Th17 cells detection, isolated peripheral blood mononuclear cells (PBMCs) were cultured at a density of 2×10^6^ cells/mL with 50ng/mL phorbol myristate acetate, 1mmol/L ionomycin (both from Sigma, St. Louis, MO, US) and 10mg/mL brefeldin A (TocrisCookson, Bristol, UK) in complete RPMI-1640 (Invitrogen, Carlsbad, CA, US) supplemented with 10% heat-inactivated fetal bovine serum (Gibco, Grand Island, NY, US) at 37°C in 5% CO2 environment for 5 hours. Upon harvest, cells were first surface-stained with PerCP-CD3 and FITC-CD4 for 20mins, fixed and permeabilized with Fix/Perm solution kit according to the manufacturer’s instructions, and then stained intracellularly with phycoerythrin PE-IL17A. For analysis of Treg cells, the whole peripheral blood samples (200ul) were first stained with PerCP-CD3, FITC-CD4 and APC-Cy7-CD25 for 20mins, then fixed and permeabilized. After permeabilization, cells were incubated with PE-FoxP3 for 30mins. Isotope controls were used to ensure antibody specificity. All labeled cells were analyzed using BD FACSCanto II.

The article "Circulating FoxP3+ Regulatory T and Interleukin17-Producing Th17 Cells Actively Influence HBV Clearance in De Novo Hepatitis B Virus Infected Patients after Orthotopic Liver Transplantation" was retracted in 2019. Reasons: missing or withdrawn patient consent; ethical violations by an author; concerns about the data.

### Enzyme linked immunosorbent assay (ELISA)

Serum levels of IL2 (Cat. #D2050), IL6 (Cat. #D6050), IL22 (Cat. #D2200) and TGF-β1 (Cat. #DB100B) were measured using ELISA kits (R&D, Minneapolis, MN, US) according to the instructions provided by the manufacturer. The sensitive for these ELISA kits were 7pg/mL, 0.7pg/mL, 5.8pg/mL and 15.4pg/mL respectively. All samples were assessed in triplicate.

### RNA isolation and RT-PCR

Total RNA was isolated from human liver biopsy using TRIZOL reagent (Invitrogen, Carlsbad, CA, US). First-strand cDNA was produced using the SuperScript II Reverse Transcriptase (Invitrogen). The first strand cDNA (1uL) was mixed with SYBR Green PCR master mix (Applied Biosystems, Foster City, CA, USA) in a final volume of 20uL. Real-time quantitative PCR was performed using 7500 Real-Time PCR System (Applied Biosystems). Primers for FoxP3 (forward: 5’-ATTCCCAGAGTTCCTCCACAAC-3’, reverse: 5’-ATTGAGTGTCCGCTGCTTCTC-3’), RORγt (forward: 5’-CAATGGAAGTGGTGCTGGTTAG-3’, reverse: 5’-TTAGGGAGTGGGAGAAGTCAAAG3’), and for glyceraldehyde 3-phosphate dehydrogenase (GAPDH) (forward: 5’- ATGAGCCCCAGCCTTCTCCAT-3’, reverse: 5’-GGTCGGAGTCAACGGATTTG-3’) were used respectively. All samples were normalized to GAPDH. Specific mRNA expression was calculated using the △△CT method.

### Immunolocalization of IL17 and FoxP3

Paraformaldehyde-fixed and paraffin-embedded human liver sections (5 mm) followed by heat mediated antigen retrieval with sodium citrate buffer (pH 6.0, 0.1mol/L) for 20mins were incubated with Anti-IL17A antibody (5μg/ml, ab136668, abcam, Cambridge, MA, US) or Anti-FOXP3 antibody (20μg/ml, ab22510, abcam) overnight at 4°C after blocking endogenous peroxidase activity with 0.3% H_2_O_2_. Revelation of primary antibody was carried out using horseradish peroxidase (HRP)-conjugated rabbit polyclonal anti-mouse (ab6728, abcam), secondary antibody followed by diamino-benzidine (DAB) and haematoxylin coloration.

### Western Blotting

Liver samples was homogenized and lysed on ice for 30mins in RIPA buffer (50mM Tris-HCl pH 7.4; 1% Triton X-100; 25mM HEPES; 150mM NaCl; 0.2% deoxycholate; 5mM MgCl_2_; 1mM Na_3_VO_4_; 1mM NaF). The tissue extract was cleared from cellular debris and nuclei by centrifugation at 10,000 rpm, and identical amounts of protein (30ug) as detected by BCA assay (Pierce, Rockford, IL, USA) were separated by Sodium Dodecy1 Sulfate-Polyacrylamide Gel Electrophoresis (SDS-PAGE) and transferred onto polyvinylidene fluoride membranes (Amersham, Little Chalfont, UK). Nonspecific binding sites were blocked with Tris-buffered saline (TBS; 40mM of Tris [pH7.6] and 300mM of NaCl) containing 5% nonfat dry milk for 2 hours at room temperature. Membranes were incubated with monoclonal anti-human FoxP3, IL17 or B-action in TBS with 0.1% Tween, and then with HRP-conjugated secondary antibodies. Immunoreactive proteins were detected by enhanced chemiluminescence and LAS-3000 imager analysis (Fujifilm Europe, Düsseldorf, Deutschland).

The article "Circulating FoxP3+ Regulatory T and Interleukin17-Producing Th17 Cells Actively Influence HBV Clearance in De Novo Hepatitis B Virus Infected Patients after Orthotopic Liver Transplantation" was retracted in 2019. Reasons: missing or withdrawn patient consent; ethical violations by an author; concerns about the data.

### Statistical analysis

Normally distributed data were expressed as x ± s, and abnormally distributed variables were described as range and median. Wald’s chi-squared test was used for categorical comparisons and continuous variables were compared using the t-test. Fisher’s exact test was used to examine the significance of any association between categorical data when the sample size was small. The Mann-Whitney non-parametric U test was used for nonparametric analyses. The Spearman’s rank correlation analysis was performed to evaluate the relationship between variables. P < 0.05 was considered to be statistically significant. SPSS 16.0 statistical software (Version 16.0, SPSS Inc., Chicago, IL, USA) was used for data analysis

## Result

### Clinical characteristics of different outcomes of DNHB-OLT Patients

The virological, serological, and clinical features of the DNHB-OLT patients were listed in Table 2. Cellular rejection was excluded by histological examination and doses of immunosuppressant (tacrolimus or mycophenolate mofetil) were not changed at the time of the De Novo HBV diagnosis. When HBV DNA was detected, LAM was started immediately for all the patients. As shown, for patient 1 and 7, tenofovir (TDF) was added to LAM therapy because of the persistent presence of HBV DNA. The remaining 10 patients received LAM monotherapy and responded very quickly. HBV DNA was undetectable in all patients at a mean of 2.67±1.23 (range = 1–5) months. Nucleotide analog was discontinued in patients in whom anti-HBs appeared and persisted (>6 months). No graft loss or fulminant hepatitis was found. The clinical courses were not uniform. After 6 months, 5 cases (patient 3, 8, 10, 11 and 12) converted into HBsAg negative and showed a resolving course with anti-HBs appearance (HBsAg seroconversion). The remaining 7 cases stayed with HBsAg positive during 6 months and HBeAg was persistently positive. The titers of HBsAb before OLT were higher in patients with HBsAg seroconversion than that with HBsAg persistence (p<0.01). HBV DNA levels ranged from 10^5^ to 10^8^ IU/mL and ALT ranged from 52 to 435 (U/L). The baseline HBV DNA, ALT levels and HBeAg status were not significantly different between patients with HBsAg seroconversion and that with HBsAg persistence respectively (p = 0.29, p = 0.07, p = 0.97). With respect to genotypes, 7 patients had genotype B, and the remaining 5 had genotype C; genotypes B and C were not related to HBsAg loss (p = 0.97).

The article "Circulating FoxP3+ Regulatory T and Interleukin17-Producing Th17 Cells Actively Influence HBV Clearance in De Novo Hepatitis B Virus Infected Patients after Orthotopic Liver Transplantation" was retracted in 2019. Reasons: missing or withdrawn patient consent; ethical violations by an author; concerns about the data.

**Table 2:** Virological, Serological, and Clinical Features of Patients with DNHB-OLT. PBC, Primary Biliary Cirrhosis; AIH, Autoimmune Hepatitis; BA, Biliary Atresia; LAM, Lamivudine; TDF, Tenofovir; Normal values: ALT, 0–40U/L; HBsAb, 0–1mIU/mL

Number	Pre-OLT		Post-OLT						
	Indication for OLT	HBsAb (mIU/mL)	Time of infection (month)	ALT (U/L)	HBVDNA (Log 10IU/mL)	HBV Genotype	HBeAg	Antiviral therapy	HBsAg clearance time (month)
1	Alcohol	+ (37.4)	9	54	7.77	B	+	LAM/TDF	no
2	HCV	- (0.2)	31	113	6.98	B	+	LAM	no
3	PBC	+(>1000)	13	327	7.96	C	-	LAM	4
4	BA	+ (64.9)	18	61	7.48	B	+	LAM	no
5	AIH	-(0.8)	23	78	7.51	C	+	LAM	no
6	Alcohol	+ (171.8)	25	391	6.87	C	+	LAM	no
7	PBC	+ (61.5)	19	52	8.03	C	+	LAM/TDF	no
8	Alcohol	+(70.4)	24	63	6.20	B	-	LAM	2
9	Alcohol	+(20.1)	22	55	7.13	C	+	LAM	no
10	Alcohol	+(617)	7	311	6.49	B	+	LAM	4
11	AIH	+(175)	16	435	7.35	B	-	LAM	3
12	BA	+(547)	15	303	7.18	B	+	LAM	2

### Serum levels of Th17 and Treg cell-related cytokines

We selected four cytokines primarily related to Th17 and Treg cells differentiation to study about the differentiation environment in different groups when diagnosed DNHB-OLT or AHB (the onset point), including interleukin-22 (IL22), interleukin-6 (IL6), transforming growth factor-beta1 (TGF-β1) and interleukin-2 (IL2). As shown in Fig 1, the levels of IL2 and TGF-β1 in DNHB-OLT group were significantly elevated compared to AHB and OLT (Fig 1C and 1D). On the contrary, the expressions of IL22 and IL6 were obviously lower than those in AHB group, but not very different with the OLT group (Fig 1A and 1B).

**Fig 1:** Serum levels of Th17 and Treg-related cytokines in different groups. IL6 (A), IL22 (B), IL2 (C), and transforming growth factor1 (TGF)-β1 (D) were tested. *P < 0.05, **P < 0.01, ***P < 0.001, **** P < 0.0001, ns p>0.05. Acute Hepatitis B Virus (AHB), De Novo Hepatitis B Virus after Orthotopic Liver Transplantation (DNHB-OLT), Control post-ttransplant cases (OLT)

### Peripheral Th17 and Treg cells frequencies

Based on our knowledge of the cytokines milieu in these patients, we analyzed the peripheral Th17 (Fig 2A) and Treg (Fig 2B) cells subsets in the total CD4+T cells population using flow cytometry at the onset point. The percentages of IL17-producing Th17 cells in DNHB-OLT (1.49 ± 0.11%) group were significantly lower than those in the AHB (3.55 ± 0.12%, P<0.0001) group, but no significant difference comparing to OLT (1.28 ± 0.14%, P = 0.274) group (Fig 2C). On the other hand, the percentages of Treg cells in the DNHB-OLT (13.61 ± 0.97%) group were significantly higher than those in the AHB (10.83 ± 0.79%, P = 0.031) and OLT (4.19 ± 0.22%, P<0.0001) groups (Fig 2D). Given the nonsynchronous changes of Treg and Th17 cells, and to better understand the relationship between these two types of immune cells, we used the ratios of Treg toTh17. Surprisingly, the ratios in the DNHB-OLT (9.31 ± 0.39%) group were significantly higher compared with the OLT (3.51% ± 0.20%, P<0.0001) and AHB groups (3.01% ± 0.14%, P<0.0001) (Fig 2E). These data indicate that a significant imbalance in the numbers of circulating CD4+T cells occurs in patients with DNHB-OLT.

The article "Circulating FoxP3+ Regulatory T and Interleukin17-Producing Th17 Cells Actively Influence HBV Clearance in De Novo Hepatitis B Virus Infected Patients after Orthotopic Liver Transplantation" was retracted in 2019. Reasons: missing or withdrawn patient consent; ethical violations by an author; concerns about the data.

**Fig 2:** Frequencies of Th17 and Treg cells, and the ratio of Treg to Th17 in the peripheral blood mononuclear cells by flow cytometry. Representative dot plots of intracellular IL17 (A) and FoxP3 (B) staining in different groups. The proportion of IL17 cells (C) and Treg cells (D) among CD4+ cells, and the ratio of Treg to Th17 (E) were shown as box plot graphs. **** P < 0.0001; *P < 0.05, ns p>0.05

### Th17 and Treg mRNA and protein expression levels in liver

To further investigate the IL17-producing Th17 and Treg cells in human liver, we also measured the gene expression by real time quantitative PCR and protein expression using immunohistochemistry and western-blot. In human liver, Th17 (Fig 3A) and Treg (Fig 3B) positive cells were distributed in CD4+ cells mainly located in portal areas with brownish-yellow color. The expressions of RORγt mRNA (Th17 cells) in the DNHB-OLT group were significantly lower than those in the AHB (P<0.0001) group, while no significant difference comparing to OLT group (P = 0.07) (Fig 3C). The expressions of FoxP3 mRNA (Treg cells) were significantly up-regulated in the DNHB-OLT liver than those in either AHB (P = 0.04) or OLT (P<0.0001) livers (Fig 3D). Next, IL17-producing Th17 (Fig 3E) and FoxP3 (Fig 3F) protein were detected by western blotting in the liver, and they had the same change tendency with the gene expressions.

**Fig 3:** Distribution and expression of Th17 and FoxP3 cells in liver. IL17 (A) and FoxP3 (B) positive cells by immunohistochemistry in DNHB-OLT patients. The gene expression of RORγt mRNA (C) and FoxP3 (D). Western- blot analysis of IL17 (E) and Treg (F).

### Clinical parameters correlation with IL17 producing Th17 cells and Treg cell frequencies

To further detect the relationship between the IL17-producing Th17 or Treg frequencies and liver injury or virus levels, we analyzed the correlations between Th17 cells or Treg cells and plasma ALT levels or HBVDNA load in these groups. As shown in Fig 4, a significantly positive correlation was only found between IL17 producing Th17 cells frequencies and ALT levels in all patients. Further analysis indicated that the positive association occurred only in the AHB patients but not the DNHB-OLT patients (Fig 4A). No correlation was found between Treg frequencies and ALT levels in any groups (Fig 4B). We also found the positive correlation between Treg frequencies and HBV DNA loads. Further analysis showed that the positive association occurred only in the DNHB-OLT patients but not in the AHB patients (Fig 4D). No correlation was found between IL17 producing Th17 cells frequencies and HBV DNA loads in any groups (Fig 4C). When all patients were divided into 2 groups based on virus clearance or non-clearance, we found that patients with virus clearance had higher IL17 producing Th17 cells (P = 0.004) (Fig 4E) and lower Treg (P = 0.31) (Fig 4F) cells than patients with the non-clearance patients, especially the sharp fall in the ratio of Treg to Th17 (P<0.0001) (Fig 4G). Thus, these results suggest that the increase of IL17 producing Th17 cells are correlated with severe liver damage in the AHB patients, which contribute to viral clearance. The increase of Treg cells are associated with poor anti-HBV immune response, leading to poor viral clearance in the DNHB-OLT patients.

The article "Circulating FoxP3+ Regulatory T and Interleukin17-Producing Th17 Cells Actively Influence HBV Clearance in De Novo Hepatitis B Virus Infected Patients after Orthotopic Liver Transplantation" was retracted in 2019. Reasons: missing or withdrawn patient consent; ethical violations by an author; concerns about the data.

**Fig 4:** Correlation between the frequencies of Th17, Treg and clinical parameters in different groups, as well as comparison of Th17, Treg, and the ratio of Treg to Th17 between clearance and non-clearance patients. Correlation IL17 with ALT (A), Treg with ALT (B), IL17 with HBVDNA (C) and Treg with HBVDNA (D) in AHB (black) and DNHB-OLT (red) patients. Furthermore, all patients were divided into 2 groups based on virus clearance. Treg (E), Th17 (F) and the ratio of Treg to Th17 (G) between clearance (black) and non-clearance (red) patients. Solid line, linear growth trend; r, correlation coefficient. *P < 0.05, **P < 0.01, ***P < 0.001, **** P < 0.0001.

### Relationship between prognosis and the Th17-Treg dynamic changes in DNHB-OLT patients

To further investigate the predictive value of the Treg, Th17 cells and the Treg to Th17 ratios in the DNHB-OLT patients, we divided DNHB-OLT patients into the clearances group in which HBsAg converted from positive to negative within 6 months and the non-clearances group in which HBsAg remain positive even after 6 months. There was no significant difference in clinical characteristics between the two groups, such as age, total bilirubin, HBV DNA and immunosuppressant (data no showed). We examined longitudinally Th17 cells, Treg cells and the ratio of Treg to Th17 dynamic changes in different groups. We observed that all patients showed distinct compositions of CD4+ cells at different times. During clearance events, the frequencies of Th17 cells displayed mild elevation during the first 4^th^ week (p = 0.072), afterwards significantly decreased from 4 to 12 weeks (p = 0.0008), and then gradually recovered back to control group (12W VS 24W, p = 0.8234; 24W VS OLT, p = 0.4871) (Fig 5A). In contrast, the Treg cells showed obviously decreased from the onset point to 12 weeks (0W VS 4W, p<0.0001; 4W VS 12W, p = 0.0002) and slightly reached control group (12W VS 24W, p = 0.7821; 24W VS OLT, p = 0.1182) (Fig 5D). The change in the ratio of Treg to Th17 had the same trend with the Treg cells (Fig 5G). During non-clearance events, the frequencies of Th17 cells remained stable (Fig 5B). However strikingly, the Treg cells reached the maximal peak during the initial 4^th^ week (p = 0.0407) and exhibited a sharply decrease from 4 to 24 weeks (4W VS 12W, p<0.0001; 12W VS 24W, p = 0.0008), then approached to the control group (p = 0.9780) (Fig 5E). The ratio also showed the consistent change tendency with Treg cells (Fig 5H).

The article "Circulating FoxP3+ Regulatory T and Interleukin17-Producing Th17 Cells Actively Influence HBV Clearance in De Novo Hepatitis B Virus Infected Patients after Orthotopic Liver Transplantation" was retracted in 2019. Reasons: missing or withdrawn patient consent; ethical violations by an author; concerns about the data.

**Fig 5:** Comparison of Th17, Treg and the ratio of Treg to Th17 between clearance and non-clearance, as well as during 24th week of follow-up in DNHB-OLT group. Treg (A), Th17 (B) and the ratio of Treg to Th17 (C) cells between clearance (black) and non-clearance (red) patients in DNHB-OLT. The dynamics of the ratio of Treg to Th17 (D, E, F) at 4th week, 12th week, and 24th week of follow-up in clearance (black) and non-clearance (red) patients and OLT (blue). *P < 0.05, **P < 0.01, ***P < 0.001, **** P < 0.0001, ns p>0.05

Compared to clearance group, the Th17 cells production at 4^th^ week was significantly lower (p = 0.0128) and the Treg cells production at 4^th^ and 12^th^ week was significantly higher (4W, p<0.0001; 12W, p = 0.001) in non-clearance group. No difference at the onset and end point (Fig 5C and 5F). However, the ratio of Treg to Th17 was significantly higher at the onset point (p = 0.0241), 4^th^ (p<0.0001) and 12^th^ (p = 0.0086) week, but the same at the end point (p = 0.4507) (Fig 5I).

## Discussion

The present study is the first report on the involvement of Treg and Th17 cells in DNHB-OLT by measuring gene, protein and T cell phenotypes in the peripheral blood and the liver. We longitudinally identified the pattern of dynamic changes in Treg and Th17 cells and demonstrated that a Treg and Th17 immune imbalance existed in DNHB-OLT patients. We found Treg frequencies and related anti-inflammatory cytokines such as IL-2 and TGF-β were significantly elevated in the DNHB-OLT patients compared to the AHB and OLT groups. And we also found IL17 frequencies and related pro-inflammatory cytokines such as IL17 and IL22 were lower in the DNHB-OLT patients than the AHB patients, but no significant difference comparing to the OLT groups in both blood level and in the liver. More importantly, we showed the Th17, Treg cells and the ratio of Treg to Th17 were associated with the HBV clearance of DNHB-OLT patients.

The article "Circulating FoxP3+ Regulatory T and Interleukin17-Producing Th17 Cells Actively Influence HBV Clearance in De Novo Hepatitis B Virus Infected Patients after Orthotopic Liver Transplantation" was retracted in 2019. Reasons: missing or withdrawn patient consent; ethical violations by an author; concerns about the data.

Immune-mediated liver injury is an important pathogenesis of HBV infection. Th17 and Treg lymphocytes cells, important subsets of CD4+ T helper cells in the cell immune function which determine the prognosis of HBV infection, play a significant role in the virus clearance and pathogenesis [20, 27, 28]. Th17 cells can enhance the capacity of mDCs and monocytes to release pro-inflammatory cytokines, which are implicated in host defense against a number of microorganisms and participate in liver tissue inflammation during hepatitis B infection [29, 30]. By contrast, Treg cells display suppressive and surveillance functions in immune responses and inflammatory diseases [31]. They not only mitigate HBV-specific immune responses but also influence innate immunity in the early phase of acute HBV infection by regulating influx of macrophages and DCs [32]. Meanwhile, they also can build an environment with immunosuppressive function through the secretion of TGF-β and IL10 to inhibit the maturing of antigen-presenting cells or endow T cells with some immunity phenotype, which is called infectious tolerance [33]. So they apparently have liver-protective functions during acute viral infection, and delay virus clearance by promoting viral immune escape and persistent infection [34]. Treg and Th17 cells are closely related to each other, sharing the same origin as well as being mutually antagonistic in function. The balance between the two cells could impact the inflammation control and autoimmune inflammation. Thus it is noteworthy that the imbalance of Treg/Th17 cells is associated not only with the pathogenesis of disease but also the severity and prognosis of disease. Many studies have demonstrated that the imbalance plays an important role in the development of various liver disease, including autoimmune liver disease, alcoholic liver disease, hepatocellular carcinoma, and acute or chronic virus-associated (HBV, HCV, HEV) liver disease in humans and mice [23–25, 30, 35–41]. In our study, we found that the percentage of Treg cells, expression of FoxP3 mRNA and related anti-inflammatory cytokines such as IL2 and TGF-β in DNVH-OLT group were significantly higher than that of AHB and OLT groups. The percentage of Th17 cells, expression of RORγt mRNA and related pro-inflammatory cytokines such as IL17 and IL22 were significantly lower than that in HBV group, but without differences comparing to the OLT group. The ratios of Treg to Th17 were significantly higher compared to OLT and AHB groups. These results suggest that more Treg cells than Th17 cells were produced and the immune imbalance of Treg/Th17 existed in DNHB-OLT patients by PBMC, gene and protein level in blood and liver. Compared with OLT and AHB patients, the differentiation environment was conducive to Treg cells differentiation in DNHB-OLT patients, which were likely to chronicity after HBV infection than AHB.

The article "Circulating FoxP3+ Regulatory T and Interleukin17-Producing Th17 Cells Actively Influence HBV Clearance in De Novo Hepatitis B Virus Infected Patients after Orthotopic Liver Transplantation" was retracted in 2019. Reasons: missing or withdrawn patient consent; ethical violations by an author; concerns about the data.

Furthermore, we studied the relationship between the two types of T cells and clinical parameters, using ALT to evaluate liver inflammation, HBV DNA to evaluate virus level and virus clearance or non-clearance to evaluate disease outcome. We found that in all patients, the frequencies of IL17 and Treg correlated with ALT and HBV DNA positively respectively, but Treg had significantly correlated with HBV DNA only in DNHB-OLT patients and IL17 had significantly correlated with ALT only in AHB patients. When all patients were divided into 2 groups based on virus clearance or non-clearance, patients with virus clearance were found to have higher IL17 and lower Treg than the non-clearance patients, especially the sharp fall in the ratio of Treg to Th17. Thus, these results suggest that the increase of IL17 is correlated with severe liver damage in the AHB patients, which contribute to viral clearance. The increase of Treg is associated with poor anti-HBV immune response, leading to poor viral clearance in the DNHB-OLT patients. Th17 cells are a potential marker for the degree of liver injury, whereas Treg cells may contribute to the suppression of HBV DNA clearance. We also showed the immune imbalance ratio of Treg to Th17 correlated with virus clearance after the HBV infection. Interestingly in DNHB-OLT patients, the level of IL-17 was same with OLT controls and ALT was much lower than AHB. As we previously reported, the majority of biopsies from the HBV recurrence patients after OLT showed minimal inflammatory changes [42]. We hypothesize that host-virus-immune interactions are modified by two important factors in LT patients. First, immunosuppressive therapy may enhance HBV replication and viral protein expression in the liver, modulating host immune reactions of liver graft damage. Second, liver graft damage after viral infection is unlikely to involve human leukocyte antigen (HLA) class 1-restricted cytotoxic T lymphocyte recognition of viral gene products on infected hepatocytes because successful LT does not require HLA matching between donor and recipient.

The article "Circulating FoxP3+ Regulatory T and Interleukin17-Producing Th17 Cells Actively Influence HBV Clearance in De Novo Hepatitis B Virus Infected Patients after Orthotopic Liver Transplantation" was retracted in 2019. Reasons: missing or withdrawn patient consent; ethical violations by an author; concerns about the data.

The use of HBsAg-/HBcAb+ donors carries a risk for the potential development of de novo HBV due to latent virus or low-level replication that can be reactivated in the setting of immunosuppression [43–44], especially in HBsAg-/HBcAb- patients [5, 45]. The presence of HBsAb before LT decreases, but does not eliminate, the risk of de novo HBV. Thus, the use of HBIG, alone or in combination with LAM, should been considered for the prevention of de novo HBV [46]. After the de novo HBV infection, clinical courses are not ominous if the patients were treated with appropriate antiviral therapy as soon as possible. However, over 40% of the patients did not show successful HBsAg seroclearance, becoming chronic HBsAg-positive carriers [7, 8]. In our study, we conducted the same results. All the DNHB-OLT patients had no graft loss or fulminant hepatitis and HBV DNA was undetectable at a mean of 2.67±1.23 (range = 1–5) months. After 6 months, 5 cases showed a resolving course with HBsAg seroconversion, whereas 7 cases stayed with HBsAg persistently positive. We longitudinally identified the pattern of dynamic changes in the Treg and Th17 cells to explore the immune pathogenesis of DNHB-OLT patients and determined their relation with their clinical outcomes after antiviral therapy. We found that the ratio of Treg to Th17 in non-clearance group was significantly higher from the onset point to 12 weeks compared to clearance group, associated with the lower Th17 cells production during the initial 4 weeks and the higher Treg cells during the 12 weeks. These data suggest that the balance between the Treg and Th17 cells at the different time pointsplays an important role during HBV clearance in DNHB-OLT patients. The higher ratios of Treg to Th17 may suppress the ability of immune clearance of the body and promote the sustained HBV replication and infection, which represent a prognostic marker for a poor virus clearance in DNHB-OLT patients.

Several previous studies have shown restoration of HBV-specific T-cells response during nucleoside analog antiviral therapy, such as LAM, Adefovir (ADV), Entcavir (ETV), is associated with CD4+ T-cells activity, which shows increase in Th17 cells and decrease in Treg cells, with significantly reduction in the ratios of the Treg to Th17 [15, 47–49]. In our study, we also observed the Th17, Treg cells and the ratios in both clearance patients and non-clearance patients were significantly lower at the end of point than those at the onset point, then approached to the control group. There were no difference in the Th17, Treg cells and the ratios among different groups at the end point. We hypnotized the effects of antiviral therapy, which directly blocked viral replication, affected Treg and Th17 cells. It seems likely that antiviral therapy result in a significant fall in the HBV DNA levels and that this in turn lead to a change in the cytokine environment, which favors a significant reduction in the ratios of Treg to Th17, together with the decrease in Treg cells and increase in Th17. It is HBV infection that results in the temporary increased Treg cells in non-clearance patients and increased Th17 cells in clearance patients during the initial 4 weeks. Therefore, with the suppression of HBV replication and the recovery of liver function, the imbalances of immune environment gradually return to the normal. These results suggest that early intervention using antiviral therapy improves the long term outcomes of DNHB-OLT patients to prevent HBV chronicity.

The article "Circulating FoxP3+ Regulatory T and Interleukin17-Producing Th17 Cells Actively Influence HBV Clearance in De Novo Hepatitis B Virus Infected Patients after Orthotopic Liver Transplantation" was retracted in 2019. Reasons: missing or withdrawn patient consent; ethical violations by an author; concerns about the data.

There are also some limitations in our present study. The chief is the limited sample population of DNHB-OLT patients in our study. Second is that peripheral blood immune responses are different from liver immune environment. For example, large Kupffer cells existing only in liver but not peripheral blood primarily release IL10 and other cytokines that can affect the differentiation and activation of CD4+ cells in liver. Therefore, the liver Treg, Th17 cells, and their cytokines’ microenvironment will be studied in our future research.

## Conclusion

In conclusion, we suggested that DNHB-OLT patients possessed a favorable Treg differentiation environment, accompanied by sustained higher preferentially Treg frequencies and up-regulation of related anti-inflammatory cytokines. The immune imbalance of the ratios between Treg and Th17 existed in DNHB-OLT patients. More importantly, we found that the ratios of Treg to Th17 in the non-clearance DNHB-OLT patients was significantly higher at the onset point, displayed an initial increase, subsequently exhibited a continuous decrease and finally approached to the normal levels. This immunosuppressive environment on one hand inhibited the inflammatory reaction of immune response, making the inflammation response in liver tissues lighter than that in AHB patients. On the other hand, this same environment suppressed the specific ability of HBV clearance, causing immune escape and chronicity easily. These findings provide new information regarding the pathogenesis of De Novo Hepatitis B Virus Infection after Orthotopic Liver Transplantation, and the ratios of Treg to Th17 may represent a potential prognostic marker for the disease.

The article "Circulating FoxP3+ Regulatory T and Interleukin17-Producing Th17 Cells Actively Influence HBV Clearance in De Novo Hepatitis B Virus Infected Patients after Orthotopic Liver Transplantation" was retracted in 2019. Reasons: missing or withdrawn patient consent; ethical violations by an author; concerns about the data.

## References

[1] ThuluvathPJ, GuidingerMK, FungJJ, JohnsonLB, RayhillSC, PelletierSJ. Liver transplantation in the United States, 1999–2008. Am J Transplant 2010; 10(pt 2):1003–1019.2042064910.1111/j.1600-6143.2010.03037.x

[2] YuL, KoepsellT, ManhartL, IoannouG. Survival after orthotopic liver transplantation: the impact of antibody against hepatitis B core antigen in the donor. Liver Transpl 2009; 15:1343–1350. 10.1002/lt.21788 19790164

[3] MerrillRM, HunterBD. Seroprevalence of markers for hepatitis B viral infection. Int J Infect Dis 2011; 15:e78–e121. 10.1016/j.ijid.2010.09.005 21130675

[4] LevreroM, PollicinoT, PetersenJ, BelloniL, RaimondoG, DandriM, et al Control of cccDNA function in hepatitis B virus infection. J Hepatol 2009; 51: 581–592. 10.1016/j.jhep.2009.05.022 19616338

[5] PrietoM. Antibody to hepatitis B core antigen-positive grafts: not perfect but no longer marginal. Liver Transpl 2009; 15: 1164–1168. 10.1002/lt.21814 19790162

[6] LaiCL, RatziuV, YuenMF, PoynardT. Viral hepatitis B. Lancet 2003; 362: 2089–2094. 1469781310.1016/S0140-6736(03)15108-2

[7] SuWJ, HoMC, NiYH, WuJF, JengYM, ChenHL, et al Clinical Course of De Novo Hepatitis B Infection After Pediatric Liver Transplantation. Liver Transplantation 2010; 16(2): 215–221. 10.1002/lt.21980 20104496

[8] BohorquezHE, CohenAJ, GirgrahN, BruceDS, CarmodyIC, JoshiS, et al Liver Transplantation in Hepatitis B Core–Negative Recipients Using Livers From Hepatitis B Core–Positive Donors: A 13-Year Experience. Liver Transplantation 2013; 19(6): 611–618. 10.1002/lt.23644 23526668

[9] LokAS, McMahonBJ. Chronic hepatitis B. Hepatology 2001; 34: 1225–1241. 1173201310.1053/jhep.2001.29401

[10] KaoJH, ChenDS. Global control of hepatitis B virus infection. Lancet Infect Dis 2002; 2: 395–403 1212735110.1016/s1473-3099(02)00315-8

[11] RehermannB, NascimbeniM. Immunology of hepatitis B virus and hepatitis C virus infection. Nat Rev Immunol 2005; 5: 215–229. 1573895210.1038/nri1573

[12] LohseAW, Weiler-NormannC, TiegsG. Immune-mediated liver injury. J Hepatol 2010; 52: 136–144. 10.1016/j.jhep.2009.10.016 19913936

[13] WangFS. Clinical immune characterization of hepatitis B virus infection and implications for immune intervention: progress and challenges. Hepatol Res 2007; 37: S339–S346. 1793118410.1111/j.1872-034X.2007.00222.x

[14] MillsKH. Regulatory T cells: friend or foe in immunity to infection? Nat Rev Immunol 2004; 4: 841–855. 1551696410.1038/nri1485

[15] FranzeseO, KennedyPT, GehringAJ, GottoJ, WilliamsR, MainiMK, et al Modulation of the CD8t-T-cell response by CD4+CD25+ regulatory T cells in patients with hepatitis B virus infection. J Virol 2005; 79: 3322–3328. 1573122610.1128/JVI.79.6.3322-3328.2005PMC1075696

The article "Circulating FoxP3+ Regulatory T and Interleukin17-Producing Th17 Cells Actively Influence HBV Clearance in De Novo Hepatitis B Virus Infected Patients after Orthotopic Liver Transplantation" was retracted in 2019. Reasons: missing or withdrawn patient consent; ethical violations by an author; concerns about the data.

[16] StoopJN, van der MolenRG, BaanCC, van der LaanLJ, KuipersEJ, KustersJG, et al Regulatory T cells contribute to the impaired immune response in patients with chronic hepatitis B virus infection. HEPATOLOGY 2005; 41: 771–778. 1579161710.1002/hep.20649

[17] Xue-SongL, Cheng-ZhongL, YingZ, Mo-BinW. Changes of treg and th17 cells balance in the development of acute and chronic hepatitis B virus infection. BMC Gastroenterol 2012; 12:43 10.1186/1471-230X-12-43 22548790PMC3404917

[18] LiJ, QiuSJ, SheWM, WangFP, GaoH, LiL, et al Significance of the balance between regulatory T (Treg) and T helper 17 (Th17) cells during hepatitis B virus related liver fibrosis. PLoS One 2012; 7 (6): e39307 10.1371/journal.pone.0039307 22745730PMC3380028

[19] SunHQ, ZhangJY, ZhangH, ZouZS, WangFS, JiaJH. Increased Th17 cells contribute to disease progression in patients with HBV-associated liver cirrhosis. J. Viral Hepat 2012; 19: 396–403. 10.1111/j.1365-2893.2011.01561.x 22571901

[20] WeaverCT, HattonRD. Interplay between the TH17 and TReg cell lineages: a (co-)evolutionary perspective. Nat Rev Immunol 2009; 9: 883–889. 10.1038/nri2660 19935807

[21] ZhouL, ChongMM, LittmanDR. Plasticity of CD4+T cell lineage differentiation. Immunity 2009; 30: 646–655. 10.1016/j.immuni.2009.05.001 19464987

[22] HooperLV, MacphersonAJ. Immune adaptations that maintain homeostasis with the intestinal microbiota. Nat. Rev. Immunol 2010; 10: 159–69. 10.1038/nri2710 20182457

[23] LiJ, ShiJ, RenW, WuW, ChenZ. Regulatory Role of CD4+CD25+Foxp3+ Regulatory T Cells on IL-17-Secreting T Cells in Chronic Hepatitis B Patients. Dig Dis Sci 2014; 59: 1475–1483. 10.1007/s10620-013-3022-1 24442238

[24] LiangXS, LiCZ, ZhouY, YinW, LiuYY, FanWH. Changes in circulating Foxp3+ regulatory T cells and interleukin-17-producing T helper cells during HBV-related acute-on-chronic liver failure. World of gastroenterology 2014; volume 20 (26): 8558–8571.10.3748/wjg.v20.i26.8558PMC409370525024610

[25] YuX, GuoR, MingD, SuM, LinC, DengY, LinZ, et al Ratios of regulatory T cells/T-helper 17 cells and transforming growth factor-β1/interleukin-17 to be associated with the development of hepatitis B virus-associated liver cirrhosis. Journal of gastroenterology and hepatology 2014; 29: 1065–1072. 10.1111/jgh.12459 24236690

[26] LenciI, TisoneG, Di PaoloD, MarcuccilliF, TariciottiL, CiottiM, et al Safety of complete and sustained prophylaxis withdrawal in patients liver-transplanted for HBV-related cirrhosis at low risk of HBV recurrence. J Hepatol 2011; 55:587–593. 10.1016/j.jhep.2010.12.036 21251938

[27] BettelliE, CarrierY, GaoW, KornT, StromTB, OukkaM, et al Reciprocal developmental pathways for the generation of pathogenic effector TH17 and regulatory T cells. Nature 2006; 441: 235–238. 1664883810.1038/nature04753

The article "Circulating FoxP3+ Regulatory T and Interleukin17-Producing Th17 Cells Actively Influence HBV Clearance in De Novo Hepatitis B Virus Infected Patients after Orthotopic Liver Transplantation" was retracted in 2019. Reasons: missing or withdrawn patient consent; ethical violations by an author; concerns about the data.

[28] MucidaD, ParkY, KimG, TurovskayaO, ScottI, KronenbergM, et al Reciprocal TH17 and regulatory T cell differentiation mediated by retinoic acid. Science 2007; 317: 256–260. 1756982510.1126/science.1145697

[29] HarringtonLE, HattonRD, ManganPR, TurnerH, MurphyTL, MurphyKM, et al Interleukin 17-producing CD4+ effector T cells develop via a lineage distinct from the T helper type 1 and 2 lineages. Nat Immunol 2005; 6: 1123–1132. 1620007010.1038/ni1254

[30] ZhangJY, ZhangZ, LinF, ZouZS, XuRN, JinL, et al Interleukin-17-producing CD4+ T cells increase with severity of liver damage in patients with chronic hepatitis B. Hepatology 2010; 51: 81–91. 10.1002/hep.23273 19842207

[31] ReinerSL. Development in motion: helper T cells at work. Cell 2007; 129: 33–36. 1741878310.1016/j.cell.2007.03.019

[32] StrossLeonhard, GuntherJohannes, GasteigerGeorg, AsenT, GrafS, AichlerM, et al Foxp3+ Regulatory T Cells Protect the Liver From Immune Damage and Compromise Virus Control During Acute Experimental Hepatitis B Virus Infection in Mice. Hepatology 2012; 56 (3): 253–257.10.1002/hep.2576522487943

[33] VignaliDA, CollisonLW, WorkmanCJ. How regulatory T cells work. Nature Reviews Immunology 2008; 8(7): 523–532. 10.1038/nri2343 18566595PMC2665249

[34] ZelinskyyG, DietzeKK, HuseckenYP, SchimmerS, NairS, WernerT, et al The regulatory T-cell response during acute retroviral infection is locally defined and controls the magnitude and duration of the virus specific cytotoxic T-cell response. Blood 2009; 114: 3199–3207. 10.1182/blood-2009-03-208736 19671923

[35] KuangDM, PengC, ZhaoQ, WuY, ChenMS, ZhengL. Activated monocytes in peritumoral stroma of hepatocellular carcinoma promote expansion of memory T helper 17 cells. Hepatology 2010; 51: 154–164. 10.1002/hep.23291 19902483

[36] LanRY, SalungaTL, TsuneyamaK, LianZX, YangGX, HsuW, et al Hepatic IL-17 responses in human and murine primary biliary cirrhosis. J Autoimmun 2009; 32: 43–51. 10.1016/j.jaut.2008.11.001 19101114PMC3225053

[37] LemmersA, MorenoC, GustotT, MaréchalR, DegréD, DemetterP, et al The interleukin-17 pathway is involved in human alcoholic liver disease. Hepatology 2009; 49: 646–657. 10.1002/hep.22680 19177575

[38] RowanAG, FletcherJM, RyanEJ, MoranB, HegartyJE, O’FarrellyC, et al Hepatitis C virus-specific Th-17cells are suppressed by virus-induced TGF-beta. J Immunol 2008; 181: 4485–4494. 1880205110.4049/jimmunol.181.7.4485

[39] YasumiY, TakikawaY, EndoR, SuzukiK. Interleukin-17 as a new marker of severity of acute hepatic injury. Hepatol Res 2007; 37: 248–254. 1739751210.1111/j.1872-034X.2007.00040.x

The article "Circulating FoxP3+ Regulatory T and Interleukin17-Producing Th17 Cells Actively Influence HBV Clearance in De Novo Hepatitis B Virus Infected Patients after Orthotopic Liver Transplantation" was retracted in 2019. Reasons: missing or withdrawn patient consent; ethical violations by an author; concerns about the data.

[40] YeY, XieX, YuJ, ZhouL, XieH, JiangG, et al Involvement of Th-17 and Th1 effector responses in patients with hepatitis B. J Clin Immunol 2010; 30: 546–555. 10.1007/s10875-010-9416-3 20393789

[41] TripathyAS, DasR, RathodSB, GuravYK, ArankalleVA. Peripheral T regulatory cells and cytokines in hepatitis E infection. Eur J Clin Microbiol Infect Dis 2012; 31: 179–184. 10.1007/s10096-011-1291-1 21598072

[42] GaoYJ, ZhangM, JinB, MengFP, MaXM, LiuZW, et al A clinical-pathological analysis of hepatitis B virus recurrence after liver transplantation in Chinese patients. Journal of Gastroenterology and Hepatology 2014; 29(3): 554–560 10.1111/jgh.12404 24117714

[43] MichalakTI, PasquinelliC, GuilhotS, ChisariFV. Hepatitis B virus persistence after recovery from acute viral hepatitis. J Clin Invest 1994; 93: 230–239. 828279210.1172/JCI116950PMC293757

[44] MarusawaH, UemotoS, HijikataM, UedaY, TanakaK, ShimotohnoK, et al Latent hepatitis B virus infection in healthy individuals with antibodies to hepatitis B core antigen. Hepatology 2000; 31: 488–495. 1065527510.1002/hep.510310232

[45] SkagenCL, JouJH, SaidA. Risk of de novo hepatitis in liver recipients from hepatitis-B core antibody-positive grafts-a systematic analysis. Clin Transplant 2011; 25: E243–E249. 10.1111/j.1399-0012.2011.01409.x 21323735

[46] UedaY, MarusawaH, EgawaH, OkamotoS, OguraY, OikeF, et al De novo activation of HBV with escape mutations from hepatitis B surface antibody after living donor liver transplantation. Antivir Ther 2011; 16: 479–487. 10.3851/IMP1771 21685535

[47] StoopJN, van der MolenRG, KuipersEJ, KustersJG, JanssenHL. Inhibition of viral replication reduces regulatory T cells and enhances the antiviral immune response in chronic hepatitis B. Virology 2007; 361: 141–148. 1718480210.1016/j.virol.2006.11.018

[48] ZhangJY, SongCH, ShiF, ZhangZ, FuJL, WangFS. Decreased ratio of Treg cells to Th17 cells correlates with HBV DNA suppression in chronic hepatitis B patients undergoing entecavir treatment. PLoS One 2010; 5: e13869 10.1371/journal.pone.0013869 21079784PMC2975625

[49] BoniC, PennaA, BertolettiA, LamonacaV, RaptiI, MissaleG, et al Transient restoration of anti-viral T cell responses induced by lamivudine therapy in chronic hepatitis B. J Hepatol 2003; 39: 595–605. 1297197110.1016/s0168-8278(03)00292-7

